The article "Retrospective Evaluation of the Effectiveness of a Synthetic Glue and a Fibrin-Based Sealant for the Prevention of Seroma Following Axillary Dissection in Breast Cancer Patients" was published in 2020. Journal: Front Oncol.

# Retrospective Evaluation of the Effectiveness of a Synthetic Glue and a Fibrin-Based Sealant for the Prevention of Seroma Following Axillary Dissection in Breast Cancer Patients

**DOI:** 10.3389/fonc.2020.01061

**Published:** 2020-07-17

**Authors:** Alessandro De Luca, Domenico Tripodi, Federico Frusone, Beatrice Leonardi, Bruna Cerbelli, Andrea Botticelli, Massimo Vergine, Vito D'Andrea, Daniele Pironi, Salvatore Sorrenti, Maria Ida Amabile

**Affiliations:** ^1^Department of Surgical Sciences, Sapienza University of Rome, Rome, Italy; ^2^Department of Medico-Surgical Sciences and Biotechnologies, Sapienza University of Rome, Rome, Italy; ^3^Department of Clinical and Molecular Medicine, Sapienza University of Rome, Rome, Italy

**Keywords:** cyanoacrylate glue, fibrin sealant, breast cancer, axillary dissection, seroma

## Abstract

**Introduction:** Seroma formation represents one of the most frequent postoperative complications of axillary dissection in breast cancer (BC) patients. We aimed to retrospectively explore the effectiveness of the intraoperative use of a synthetic cyanoacrylate glue (specifically Glubran®2) vs. the intraoperative use of a fibrin sealant (specifically Tisseel) in reducing seroma formation compared to the use of nonsealant in BC patients who underwent breast surgery and axillary dissection.

**Materials and Methods:** We conducted a retrospective, monocentric observational study on BC patients who underwent axillary dissection associated with breast surgery. The axillary dissection was completed with the application of a closed suction drain and was preceded by the application of either Glubran®2 glue or Tisseel sealant or nonsealant. We analyzed the quantity of serum drained in the first 3 postoperative days, length of hospitalization, days of permanence of axillary drain, seroma development, and presence of postoperative infection signs.

**Results:** Forty-one BC patients were considered. Based on the device used during the surgical treatment, the patients were divided into three groups: group A (17 patients), to whom suction axillary drain was applied; group B (7 patients), to whom Tisseel and axillary suction drain were applied; and group C (17 patients), to whom Glubran®2 and axillary suction drain were applied. Among the three groups, we did not find significant differences in terms of amount of serum drained in the first 3 postoperative days, length of hospitalization, and incidence of seroma. Group C maintained the axillary drain in a significantly lower number of days compared to the other two groups (*p* = 0.02); it also had a lower incidence of postoperative infections (6%) compared to group A (23%) and group B (57%) (*p* = 0.02).

The article "Retrospective Evaluation of the Effectiveness of a Synthetic Glue and a Fibrin-Based Sealant for the Prevention of Seroma Following Axillary Dissection in Breast Cancer Patients" was published in 2020. Journal: Front Oncol.

**Conclusions:** We did not find any evidence that the use of surgical glues may reduce the formation of seroma following axillary dissection in BC patients. Nevertheless, the use of cyanoacrylate glue in association with closed suction axillary drain seems to contribute to the reduction in days of axillary drain permanence and of postoperative infections, which are known factors delaying the schedule of any adjuvant oncological therapies.

## Introduction

Breast cancer (BC) surgical treatment includes conservative or demolitive procedures associated to axillary staging surgery consisting of sentinel node biopsy and/or axillary dissection (1–3). It has been shown that a frequent complication of these types of treatments is represented by seroma development (4), with a percentage ranging from 15 to 85% (5), together with infection of the surgical site and bleeding. Both breast and axillary surgery, due to the dissection of small lymphatic and blood vessels, determine the formation of a highly suitable environment for the collection of fluids, although its pathophysiological process is not completely known (6).

The seroma may lead to dehiscence of the surgical wound and necrosis of the skin flaps, further increasing the risk of infection and reoperation, as well as interfering with the recovery of upper limb mobility and delaying the start of any adjuvant therapies (4, 7). Moreover, in the case of seroma, its evacuation through repeated transcutaneous aspirations may increase patient's discomfort and delay the return to common domestic and daily activities (7).

Several techniques have been tested over time to prevent the formation of seroma, i.e., use of continuous suction drainages (8), topical application of tetracyclines (9), external compression bandages (10), and use of dissectors with ultrasound technology (11). In addition, the use of fibrin sealant has presented interesting results because of its adhesive and hemostatic properties and in part also for its potential biostimulating ability for tissue regeneration (12, 13); in particular, its combination with “quilting” sutures has been documented to significantly reduce total drainage, hospital stay, and postoperative seroma incidence in patients who underwent postmastectomy breast reconstruction with dorsal muscle flap (14). Interesting results in reducing lymphatic production and seroma development after demolitive and/or conservative breast surgery and after pelvic lymphadenectomy were also obtained using a cyanoacrylate-based synthetic surgical glue (7, 15). In particular, recently, the use of a specific type of cyanoacrylate-based synthetic adhesive, Glubran®2, developed to minimize toxic effect of cyanoacrylate glues, has been described in surgery in substitution or in addition to sutures or staples for its adhesive properties and for the potential activity in decreasing activated partial thromboplastin time, exerting a hemostatic effect and therefore further contributing to tissue adhesion (16–18).

The article "Retrospective Evaluation of the Effectiveness of a Synthetic Glue and a Fibrin-Based Sealant for the Prevention of Seroma Following Axillary Dissection in Breast Cancer Patients" was published in 2020. Journal: Front Oncol.

In this light, we aimed to retrospectively explore the effectiveness of the intraoperative use of a synthetic cyanoacrylate glue (specifically Glubran®2) vs. the intraoperative use of a fibrin sealant (specifically Tisseel) in reducing seroma formation compared to the use of nonsealant in BC patients who underwent breast surgery and axillary dissection.

## Materials and Methods

### Patients

This is a retrospective, monocentric study conducted on patients diagnosed with BC and treated at the Department of Surgical Sciences, Sapienza University of Rome. The study was approved by the local Ethics Committee. All procedures were in accordance with the ethical standards of the Helsinki Declaration issued in 1975 and later amendments. We considered patients who underwent axillary dissection associated with mastectomy or breast conservative surgery. The surgical indication to axillary dissection was placed during the multidisciplinary meeting in patients with clinically positive axillary lymph nodes and cytological exam, following lymph node aspiration, positive for neoplastic cells, or in cases of sentinel node biopsy positive for the presence of macrometastasis.

The following clinical data were collected:

- age, weight, height, body mass index (BMI);
- immunohistochemical features of the tumor, radiological staging of axillary lymph nodes, eventual neoadjuvant chemotherapy performed, type of surgery performed, tumor–nodes–metastasis (TNM) staging, number of lymph nodes removed;
- length of hospital stay, daily volume of the drain content during the days of hospitalization, number of days of drain permanence at the surgical site, eventual seroma development and its aspiration, fever, infection, and/or dehiscence of the surgical wound.

### Surgical Procedure

The patients underwent surgery under general anesthesia. During axillary lymph nodes dissection, the lymphatic vessels afferent to the removed lymph nodes were tied, and the long and thoracodorsal thoracic nerves were preserved. Clips and electrocautery were used to achieve hemostasis and lymphostasis. Once the axillary lymph nodes were removed and hemostasis performed, the surgical procedure was completed with the position of a suction drain preceded by the application of a fibrin sealant (Tisseel, 2 ml), nebulized on the surgical site, or by the application of a cyanoacrylate glue (Glubran®2, 1 ml), nebulized with a dedicated system on the surgical site. There were cases conducted only with the suction drain position without the application of any sealant. The wound was then medicated and an elastocompression bandage performed.

The article "Retrospective Evaluation of the Effectiveness of a Synthetic Glue and a Fibrin-Based Sealant for the Prevention of Seroma Following Axillary Dissection in Breast Cancer Patients" was published in 2020. Journal: Front Oncol.

### Fibrin Sealant and Synthetic Cyanoacrylate Glue

Tisseel low-dose fibrin sealant, a human-derived local hemostatic drug consisting of a solution of two components, human fibrinogen, and human thrombin, was sprayed on all visible surgical surfaces in a thin layer. Contraidnications to the use of fibrin sealant were hypersensitivity to the components or to any of the excipients and intravascular use.

The Glubran®2 glue, a surgical cyanoacrylate glue of synthetic origin (combination of n-butyl cyanoacrylate and methacryloxysulfolane monomers) for internal and endovascular use, was nebulized in a small amount on the surgical site with a dedicated pressure regulator system to allow its application on all visible surfaces in a thin layer. Contraindications to the use of cyanoacrylate adhesive were hypersensitivity of the subjects to the components or to any of the excipients, and pregnancy.

### Postoperative Period Care

The compressive bandage was removed after 48 h, and patients were discharged in the second to third postoperative day, except in cases of complications and/or comorbidities.

Suction drain was checked and emptied daily during hospitalization, and the amount of serum collected was recorded. Following discharge, the patients were reviewed in an outpatient setting and the quantity of drained serum measured.

The drain was removed when the quantity of serum collected was <40 ml/day. In case of axillary seroma development after removal of the drain, its aspiration was evaluated and recorded. The decision to aspirate a seroma was based on the assessment of its volume and the discomfort reported by the patient.

Local or general signs of infection was also assessed and antibiotic therapy prescribed as needed.

### Statistical Analysis

Data regarding the quantity of serum drained in the first 3 postoperative days, duration of hospitalization, days of permanence of axillary drainage, development of seroma, and presence of signs of infection were collected. Patients' characteristics were described using mean ± standard deviation (SD) for continuous normally distributed variables.

For the comparison between groups, one-way ANOVA test was used for continuous variables and the chi-square test for categorical variables.

A *p* < 0.05 was considered statistically significant. The statistical analysis was performed with IBM SPSS Statistics 25.

## Results

### Patients' Characteristics

Forty-one BC patients who underwent axillary dissection associated with mastectomy or breast conservative surgery were considered.

The article "Retrospective Evaluation of the Effectiveness of a Synthetic Glue and a Fibrin-Based Sealant for the Prevention of Seroma Following Axillary Dissection in Breast Cancer Patients" was published in 2020. Journal: Front Oncol.

All patients received diagnosis of invasive ductal or lobular BC obtained by radiological guided breast needle biopsy.

Based on the device used during the surgical treatment, the patients were divided into three groups:

- group A, consisting of 17 patients, to whom axillary closed suction drain had been placed in the axillary fossa;
- group B, consisting of 7 patients, to whom Tisseel sealant and axillary closed suction drain had been placed in the axillary fossa;
- group C, consisting of 17 patients, to whom Glubran®2 glue and axillary closed suction drain had been placed in the axillary fossa.

The mean age of the patients was 58 ± 14.2 years, and the mean BMI was 25 ± 4.86. Patients' characteristics of each group are shown in the Table 1. Ten patients had diabetes mellitus, and 16 patients reported dyslipidemia in past medical history.

**Table 1:** Patients' characteristics.

**Breast cancer patients**	**Group A**	**Group B**	**Group C**
***N* = 41**	***N* = 17**	***N* = 7**	***N* = 17**
Age, years	55.8 ± 13.5	55.7 ± 16.2	59.1 ± 13.2
BMI, kg/m^2^	24.6 ± 4.7	25.4 ± 4.01	25.3 ± 5.4
Dyslipidemia	5	2	9
Diabetes mellitus	5	1	4
Type of surgery			
Mastectomy + AD	12	7	14
BCS + AD	5	0	3
Tumor size, cm	2.1 ± 1.2	2.4 ± 1.6	1.9 ± 1.2
Number of lymph nodes removed	11.9 ± 6.9	13 ± 6.8	8.9 ± 4.9
Number of metastatic lymph nodes	3.2 ± 1.6	5.1 ± 7.2	2.1 ± 1.4
Neoadjuvant chemotherapy	4	1	9^*^
Hystological subtype			
Ductal invasive carcinoma	13	6	15
Lobular invasive carcinoma	3	1	2
Metaplastic carcinoma	1	0	0
Immunoistochemical subtype			
Luminal A	5	4	7
Luminal B	9	1	5
Triple negative	2	1	3
Her2 enriched	1	1	2

*Data are shown as mean ± SD and n*.

*AD, axillary dissection; BCS, breast conservative surgery*.

* *P ≤ 0.05*.

The BC definitive histological diagnosis was laid for ductal invasive carcinoma in 83% of the patients, lobular invasive carcinoma in 14.6%, and metaplastic carcinoma in 2.4% (one case) (Table 1).

The average size of the breast tumor was 2.1 cm, with a maximum of 5.5 cm and a minimum of 1 cm. The most frequent immunohistochemical subtype was luminal A (39%), followed by luminal B (36.6%); the 14.6% presented a triple negative BC, and 9.7% had a Her2-enriched BC (Table 1).

The three groups were comparable in terms of age, BMI, and type of breast surgery. However, there was a higher proportion of patients who received neoadjuvant chemotherapy in group C (52%) compared to group A (18%) and group C (52%) (*p* = 0.048; Table 1). Eighty percent of the entire cohort had undergone mastectomy and axillary dissection, while 20% had undergone breast conservative surgery and axillary dissection.

The article "Retrospective Evaluation of the Effectiveness of a Synthetic Glue and a Fibrin-Based Sealant for the Prevention of Seroma Following Axillary Dissection in Breast Cancer Patients" was published in 2020. Journal: Front Oncol.

The median number of lymph nodes removed was 12 (with a maximum of 27 and a minimum of 3).

### Postoperative Course

No significant differences were documented among the three groups in terms of total amount of serum drained by the axillary drain within the first 3 postoperative days, and similarly, there was no difference in terms of mean length of hospitalization between patients in the three different groups (Table 2).

**Table 2:** Postoperative course.

**Breast cancer patients**	**Group A**	**Group B**	**Group C**	***P***
***N* = 41**	***N* = 17**	***N* = 7**	***N* = 17**	
Serum quantity drained during the first 3 postoperative days, ml	229.1 ± 124.2	261.4 ± 132.04	205.8 ± 123.9	0.77
Length of hospitalization, days	4.76 ± 0.56	4.57 ± 0.8	5 ± 0.71	0.41
Axillary drain permanence, days	14.1 ± 8.7	11.4 ± 7.9	7.4 ± 3.2	0.02
Postoperative seroma incidence, %	11.8	14	6	0.76
Incidence of postoperative infections, %	23	57	6	0.02

When considering the total number of days of the axillary drain maintained at the surgical site, we observed a significant difference among the three groups (*p* = 0.02; Table 2). In group C, we observed a lower number of days of drain (7 days) compared to group A (14 days) and group B (11 days; Table 2).

The incidence of postoperative seroma was 11.8% in group A, 14% in group B, and 6% in group C (*p* = 0.76; Table 2).

Interestingly, signs of postoperative infection were significantly lower in group C compared to that in the other two groups (*p* = 0.02; 23% of patients in group A, 57% of group B, and 6% of group C) (Table 2).

Considering the known contribution of a high BMI to an increased potential seroma formation (7), we have additionally investigated a possible correlation between patients' BMI and the total days of permanence of axillary drain, as well as between patients' BMI and quantity of serum drained in the first 3 postoperative days, but we did not find any significant positive correlation either in all the enrolled participants either in each group of participants.

## Discussion

In our study, we observed that, although the use of two different surgical sealants was not associated with a reduction in the incidence of postoperative seroma, the use of cyanoacrylate glue has led to a reduced occurrence of postoperative infections and has allowed a short time of permanence of the axillary drain, maintaining an incidence of seroma development similar to that of the group where no sealant was applied and the drain maintained in the surgical site at least twice the number of days.

The reduction in terms of number of days for the permanence of the axillary drain is certainly beneficial for patients. First, its presence implies the need for repeated outpatient controls. Second, it affects patient's mobility since its location within the surgical wound can give pain and limit movements of the upper limb involved. Moreover, it may also happen that, due to eventual abrupt movements of the limb, the drainage is unknowingly dislocated, causing pain and worry to the patient.

The article "Retrospective Evaluation of the Effectiveness of a Synthetic Glue and a Fibrin-Based Sealant for the Prevention of Seroma Following Axillary Dissection in Breast Cancer Patients" was published in 2020. Journal: Front Oncol.

It is also important to consider that any adjuvant therapies (chemotherapy and/or radiotherapy) can be started only when the surgical wound has completely healed; therefore, the permanence of axillary drainage might delay its scheduling (19). In this light, for cancer patients, reducing the rate and duration of complications in the postoperative period represents certainly an advantage.

Similar to the results obtained by Vasileiadou et al. (7), our findings may be in part explained by the fact that the Glubran®2 rapidly polymerizes into a thin elastic film, which presents elevated tensile strength and adheres to the tissue once applied. Consequently, the use of this cyanoacrylate glue during surgery may create a sealing coating, which can prevent or reduce seroma formation likely due to a better approximation of wound margins, resulting in a smaller dead volume, and determining a potentially more permanent effect on tissues with respect to the fibrin sealant (12). Cyanoacrylate glue is potentially cytotoxic (20), and it has to be highlighted the importance of training in its application, choosing the right application device, which, for the prevention/treatment of axillary lymphorrhea, consists in nebulizing a small amount of glue through a dedicated nebulizer system in the operating field.

Our study focuses on seroma prevention techniques after axillary dissection, given the relevance of this type of surgery to date. In fact, despite the tendency of BC surgery to an increasingly conservative approach, axillary lymphadenectomy remains an essential intervention in several clinical settings to complete the disease staging (21): in the presence of clinically pathological axillary lymph nodes; in case of preoperative cytological study of lymph nodes with finding of metastatic cells; in the presence of sentinel lymph node histologically positive for macrometastasis; in T4 tumors and inflammatory BC (22); and in case of persistently positive axillary clinical exam following neoadjuvant therapy (21).

Axillary lymphadenectomy may cause several complications, among which the most frequent are seroma, bleeding, and surgical wound infection development (23, 24), delaying patient's recovery and any eventual adjuvant therapy. In addition, seroma may lead to limitation in upper limb movements and by postoperative pain (23, 24).

The article "Retrospective Evaluation of the Effectiveness of a Synthetic Glue and a Fibrin-Based Sealant for the Prevention of Seroma Following Axillary Dissection in Breast Cancer Patients" was published in 2020. Journal: Front Oncol.

In postoperative seroma classification, three degrees are recognized (25): (i) first degree, seroma asymptomatic, evaluable only by ultrasound exam; (ii) second degree, seroma symptomatic that requires outpatient needle aspiration; and (iii) third degree, seroma symptomatic that needs surgical and/or radiological-guided drainage. The pathogenesis of seroma is not yet well-known. Serum accumulates to fill the cavities that are inevitably created following surgical treatment as what happens in lymphadenectomy. Some authors hypothesized that an inflammatory process intervenes in the pathogenesis of seroma, which would result from the damage to vessels and tissues perpetuated during the intervention (19). Seroma may result also as an accumulation of lymph fluids resulting from the lymph nodes dissection (26). Unalp and Onal (27) have investigated the association between seroma development and type of surgery performed, as well as patient's age, weight and comorbidities, and breast volume. The authors found that a drainage flowrate of >50 ml/day after 48 h following breast surgery resulted a predicting factor for seroma formation in BC patients, while other investigated variables were not associated with development of seroma (27). Although a significant contribution of a high BMI to increased seroma formation in breast surgery (7) has been reported, a systematic review, conducted to estimate individual risk of seroma formation in breast surgery, found only moderate evidence to support a risk for seroma formation in subjects with higher body weight, extended radical mastectomy as compared with simple mastectomy, and greater drainage volume in the initial postoperative 3 days, but no risk factor to support strong evidence (28).

Regarding the use and management of suction axillary drain in patients undergoing lymphadenectomy, this topic is widely discussed in the literature, but there is no agreement between the numerous experiences. Several studies encourage the use of suction drains and advise against their early removal (before the third postoperative day) (29). A systematic review of randomized controlled trials, which involved 585 BC patients, assessed the incidence of seroma between two groups of patients who underwent axillary dissection, one treated with axillary drain position, and the other one without it (30). The incidence of postoperative seroma was 46.8% in the first group and 68.8% in the second group. The review showed that the insertion of a suction drain after axillary dissection reduced seroma development, its incidence, and the frequency of subsequent aspirations (30). On the other hand, this method increases the hospitalization length, even if experiences of early discharge with onsite drain and its outpatient management have been described. These data have been confirmed by a Cochrane review of randomized controlled trials involving 960 patients undergoing axillary dissection, with or without drain insertion (31). Ten Wolde et al. in 2014 (32) proposed, as an alternative to the use of drains following mastectomy, the use of the quilting suture, consisting in the mechanical occlusion of space through sutures along the surgical site that secure the subcutaneous tissue to the pectoral and/or dentate muscle fascia. This technique, by reducing dead spaces, resulted in the effective prevention of seroma (32). Garbay et al. described the use of quilting sutures also following axillary dissection (33). The authors observed a reduction in terms of average length of hospitalization, need for seroma aspiration, and intensity of postoperative pain (33). It has also been described by Mazouni et al. (34) the use of quilting sutures in association with suction drain for the prevention of postmastectomy seroma, which resulted in a reduction in the rate of postoperative seroma development, volume of drained seroma, and length of drain maintenance in the surgical site.

The article "Retrospective Evaluation of the Effectiveness of a Synthetic Glue and a Fibrin-Based Sealant for the Prevention of Seroma Following Axillary Dissection in Breast Cancer Patients" was published in 2020. Journal: Front Oncol.

The use of fibrin sealant as hemostatic agents in surgery is well-documented, although there are controversial results on its ability to reduce fluid accumulation in dissected spaces through tissue adhesion, as in inguinal hernia repair (35). Fibrin sealants are biological hemostatic agents that interact with tissues during surgery, promoting hemostasis, growth, and duplication of fibroblasts, and favoring closure of lymphatic vessels. Furthermore, fibrin sealant likely may mechanically obliterate the dead space where serous fluid accumulates after surgical dissection (4). Nevertheless, some studies have evaluated the use of fibrin sealant in addition (36) or in replacement (4) to the drain position, resulting in a lower hospital stay length and lower costs but not modifying significantly the incidence of postoperative seroma in the group of patients treated with fibrin sealant. Similarly, Burak et al. (37) and Langer et al. (38) documented no difference in the incidence of seroma after axillary lymph nodes dissection when using this agent, in accordance with our results. It has been hypothesized that cyanoacrylate adhesive glue may have longer and more permanent effect on tissues than the frequently used fibrin sealant, due to its properties (7). The use of cyanoacrylate glue has been described in general and laparoscopic surgery. Good results have been obtained in the treatment of acute bleeding of gastric (16) and esophageal varices (17), for the treatment of external pancreatic fistulas (39), and for mesh fixation during laparoscopic inguinal hernioplasty (18). The use of cyanoacrylate has also been evaluated in the prevention of postoperative lymphocele after lymphadenectomy in patients with uterine tumor (15), showing that in the cyanoacrylate group, only 15% of the patients developed lymphocele vs. 36% in the control group. The volume of lymphorrhea was lower in the cyanoacrylate group with respect to the control group (15). Vasileiadou et al. (7) obtained interesting results using the cyanoacrylate glue in association with the suction drainage: it seemed to contribute to the reduction in the onset of seroma, with a lower need for evacuative punctures and a reduction in terms of number of permanence days of the axillary drain. The assumed mechanism of action is that its adhesive property may create a sealing coating in the surgical field, occluding lymphatic leaks and limiting the accumulation of seroma (7), determining potential positive effects.

The article "Retrospective Evaluation of the Effectiveness of a Synthetic Glue and a Fibrin-Based Sealant for the Prevention of Seroma Following Axillary Dissection in Breast Cancer Patients" was published in 2020. Journal: Front Oncol.

Considering the results of our study, some limitations have to be acknowledged. We conducted a retrospective study, with access only to clinical data that are normally collected within routine clinical practice and with lack of methodological rigor; in fact, the sample size in the different groups was not homogeneous, with fewer patients in group B compared to groups A and C. Moreover, in group B, the presence of axillary suction drain might have compromised the stabilization of fibrin clots provided by the fibrin sealant and have interfered with adherence between tissues. Also in this setting, choosing the right spray during training for its application is important. The greater obstacle when using fibrin sealant is the mode of application in order to allow adequate activation of the glue and reach the solid phase.

In our retrospective evaluation, we found no evidence that the use of surgical glues might actually reduce the formation of seroma following axillary dissection, and in this light, each group size did not allow a reliable conclusion on this aspect.

However, we have been able to observe that the use of cyanoacrylate glue in association with the positioning of an axillary closed suction drain in patients undergoing axillary dissection may contribute to the reduction in the length of drain permanence and the incidence of infections in the postoperative period.

It would be interesting to deepen our experience by conducting further prospective and multicenter studies in this regard.

## Data Availability Statement

The raw data supporting the conclusions of this article will be made available by the authors, without undue reservation.

The article "Retrospective Evaluation of the Effectiveness of a Synthetic Glue and a Fibrin-Based Sealant for the Prevention of Seroma Following Axillary Dissection in Breast Cancer Patients" was published in 2020. Journal: Front Oncol.

## Ethics Statement

The studies involving human participants were reviewed and approved by Comitato Etico dell'Università “Sapienza,” AOU Policlinico Umberto I, Rome, Italy. The patients/participants provided their written informed consent to participate in this study.

## Author Contributions

AD and DT conducted research, analyzed data, and wrote the paper. FF conducted research. BL conducted research and analyzed data. BC, AB, MV, VD'A, and DP reviewed the paper. SS wrote and reviewed the paper. MA designed and conducted the research and wrote and reviewed the paper. All authors read and approved the final manuscript.

## Conflict of Interest

The authors declare that the research was conducted in the absence of any commercial or financial relationships that could be construed as a potential conflict of interest. The handling editor declared a shared affiliation with the authors.
